The article "Mechanisms of Intervertebral Disc Degeneration Treatment with Deer Antlers Based on Network Pharmacology and Molecular Docking" was published in 2022. Journal: Evid Based Complement Alternat Med.

# Mechanisms of Intervertebral Disc Degeneration Treatment with Deer Antlers Based on Network Pharmacology and Molecular Docking

**DOI:** 10.1155/2022/8092848

**Published:** 2022-09-06

**Authors:** Rui Weng, Hongheng Lin, Zhuoyao Li, Daman Chen, Xiaoxiao Lin, Zhenyu Zhang, Qiqi Chen, Yiqi Yao, Wenchao Li

**Affiliations:** ^1^The Third Affiliated Hospital of Guangzhou University of Chinese Medicine, Guangzhou 510375, Guangdong, China; ^2^Guangdong Research Institute for Orthopedics and Traumatology of Chinese Medicine, Guangzhou 510375, Guangdong, China; ^3^Guangzhou University of Chinese Medicine, Guangzhou 510405, Guangdong, China

## Abstract

**Background:**

With the aging of the population, the prevalence of IVDD increases preoperatively. How to better treat IVDD has become an important clinical issue. Deer antlers proved to have a great effect on the treatment of IVDD in many studies, but the molecular mechanism has not been clarified.

**Objective:**

To investigate the molecular mechanism and target of deer antlers in the treatment of IVDD.

**Methods:**

Compounds from deer antlers were collected and targets were predicted using HERB, TCMSP, TCMID, SwissADME, and SwissTargetPrediction. Collection of disease targets for IVDD was done using GeneCards, TTD, DrugBank, DisGeNET, and OMIM. Cytoscape 3.7.2, AutoDock Vina (v1.1.2), and R software were used for data analysis and the construction of network diagrams.

**Results:**

A total of 5 active compounds from deer antlers were screened and 104 therapeutic targets were predicted. A total of 1023 IVDD disease targets were collected. Subsequently, PPI network prediction analysis was performed for disease and treatment targets, and 112 core targets were collected after screening. After obtaining the core target, we used the clusterProfiler software package of R software to carry out GO and KEGG enrichment analyses for the core target and plot the bubble maps. According to the GO enrichment results, the main biological processes of IVDD treatment by deer antlers lie in the rhythmic process, mRNA catabolic process, and G1/S transition of the mitotic cell cycle. KEGG results were mainly related to the PI3K-Akt signaling pathway, thyroid hormone signaling pathway, and Notch signaling pathway. Molecular docking results showed that estrone had the best docking results on ESR1.

**Conclusion:**

Deer antlers are rich in various compounds that can prevent the development of IVDD by upregulating the PI3K-Akt signaling pathway and Notch signaling pathway. Its key compounds estradiol and estrone can reduce the inflammatory response and oxidative stress in tissues and organs, thus slowing down the progression of IVDD. Estrone, the active compound in deer antlers, was found by molecular docking to have good results against ESR1, the target of the disease, which may be a potential site for drug therapy.

## 1. Introduction

Deer antlers (Cervi Cornu Pantotrichum) refer to the outgrowths on the forehead of the male of sika deer and red deer, which are covered with a layer of velvety fur [1]. Deer antlers, owning a beneficial effect of tonifying “kidney-yang,” are normally used to treat low back pain, soreness of the knee, morbid vaginal discharge, and so on [2]. The efficiency of deer antlers is dependent on their bioactive components. Recent studies reported that the deer antlers' significant ingredients are polysaccharides, polypeptides, and free amino acids [3]. The nucleus pulposus, cartilage endplates, and annulus fibrosus constitute the intervertebral disc, which can keep the spine stable and flexible [4]. One of the main factors contributing to low back pain is intervertebral disc degeneration (IVDD) [5]. With the aging of the population, the prevalence of IVDD is increasing in proportion [6]. One study showed that the incidence of IVDD in the whole lumbar spine was 31.6% in men and 44.7% in women [7]. People have thought that inflammation and oxidative stress are closely related to IVDD. Polysaccharides have good antioxidant properties [8]. Furthermore, deer antler peptide, exhibiting significant anti-inflammatory and antioxidative effects, can effectively protect osteoblasts [9–11]. Meanwhile, proteins contained in deer antlers protect against oxidative stress and inflammation [3, 12].

Network pharmacology, which is based on the concept of a multilevel and multiangle interaction network among diseases, genes, targets, and drugs, can observe the interventional mechanism and influence of drugs on the disease network systematically and comprehensively [13]. It can generate complex networks of interactions according to target molecules, biological functions, and bioactive compounds to clarify the mechanism of action of TCM prescriptions at the molecular level [14]. Up to now, network pharmacology has been used in many studies of Chinese herbal medicine and its preparations [15]. Molecular docking is an effective tool in structural molecular biology and computer-assisted drug design that predicts a ligand's major binding mode(s) with a target protein [16]. Due to the unique therapeutic properties, deer antlers have attracted much research interest. So far, nevertheless, the target and mechanism of deer antlers in the treatment of IVDD have not been elucidated in the literature, and people know little about it, which limits the further development and application of deer antlers to some extent. This study aims to explore the potential mechanism of deer antlers action from the perspective of network pharmacology.

## 2. Materials and Methods

### 2.1. Component-Target Network

We searched for active ingredients in deer antlers using HERB (https://herb.ac.cn/), TCMSP (https://tcmsp-e.com/), TCMID (https://47.100.169.139/tcmid/), and other Chinese medicine database platforms as well as the literature. Immediately afterward, the collected active ingredients were screened for ADME on the SwissADME (https://www.swissadme.ch/index.php) using the following criteria: “GI absorption” as “HIGH” and “YES” for any two of the “Drug-likeness” cells. After obtaining the screened active ingredients from the antlers, they were imported into SwissTargetPrediction to predict the drug targets, and those with *P* values >0 were selected, validated, and supplemented in the UniProt database.

### 2.2. IVDD Target Collection

Disease-related genes were searched for in GeneCards, TTD, DrugBank, DisGeNET, OMIM, and other disease target databases using “IVDD” as the search term and screened for human race. Subsequently, the collected disease targets were aggregated and deduplicated, and they were standardized and supplemented with gene names in the UniProt database.

### 2.3. Core Target Screening

Using the BisoGenet plug-in in Cytoscape 3.7.2, protein interaction networks were predicted separately for drug component targets and disease targets, and the two networks were merged to collect their intersecting targets. Next, the CytoNCA plug-in was used to analyze the topology of the intersection network and extract the HUB targets based on the values of “Betweenness,” “Degree,” and “Closeness” in the results as filtering criteria.

### 2.4. GO and KEGG Enrichment Analyses

GO enrichment analysis is able to discover the link between genes and gene product features across all species. KEGG enrichment analysis is useful in clarifying in vivo comprehensive inferences of reactions. The R software packages “pathview” and “clusterProfiler” were used for KEGG and GO enrichment analyses of intersection targets. Finally, the “ggplot” software package was used to visualize the results.

### 2.5. Molecular Docking

Five core target proteins in the PPI network and significant components in the “component-target” network diagram were selected for molecular docking verification. The 3D structures of the target protein were downloaded from the PDB website (https://www.rcsb.org/), and the 3D structures of the components were obtained from the ZINC website (https://zinc.docking.org/). First, the intrinsic small ligand of the protein was docked to the protein structure, and the binding energy was calculated. Second, the target proteins and components were docked in AutoDock Vina (v1.1.2), and the binding energy was also calculated. The binding energy of the intrinsic small ligand to the protein was the standard for verifying the binding conditions of the new compounds. Ultimately, PyMOL (v2.5) was utilized to present a visual analysis of the molecular structure.  Figure 1 shows the brief flowchart with network pharmacology and molecular docking.

## 3. Result

### 3.1. Component-Target Network Diagram Construction

A total of 5 active ingredients were obtained from the screening of deer antlers (Table 1). A total of 104 targets were obtained after aggregation and deweighting. The data were imported into Cytoscape 3.7.2 to construct a “component-target” network diagram, which showed a total of 104 nodes and 238 component-target interactions (Figure 2). From the figure, we can find that alpha-estradiol and 17-beta-estradiol interact with the most target genes and are potential key compounds. Based on the results of the topological analysis, we attained the degree values for the five active ingredients (Table 2).

### 3.2. Results of the Core Target Screening

A total of 1023 disease targets were obtained after the search summary, and after intersection mapping with drug action targets, the intersection network was topologically analyzed using the CytoNCA plug-in. Subsequently, the “Degree” value in the results was used as a filtering criterion to screen targets with a “Degree” value greater than or equal to 2 times the median (degree ≥68), and a total of 2579 targets were obtained, that is, because the degree value can reflect the importance degree of a compound in deer antlers. Afterward, the new results were analyzed according to the three indicators “Betweenness,” “Degree,” and “Closeness,” and targets greater than or equal to the median were screened, resulting in 112 core targets (Figure 3, Table 3).

### 3.3. GO and KEGG Enrichment Analyses Results

A total of 1061 GO entries were obtained after enrichment, containing biological process (BP), cellular component (CC), and molecular function (MF), with a *P* value screening for each component. The main results are the rhythmic process, mRNA catabolic process, and G1/S transition of the mitotic cell cycle (Figures 4–6). Meanwhile, the core targets were subjected to the KEGG pathway enrichment analysis to screen for pathways with *P* < 0.05, and a total of six were obtained, such as the PI3K-Akt signaling pathway, the thyroid hormone signaling pathway, the Notch signaling pathway, the FoxO signaling pathway, the estrogen signaling pathway, and the HIF-1 signaling pathway (Figure 7), among which the specific mechanism of deer antler treating intervertebral disc degeneration in the PI3K-AKT signaling pathway is shown in Figure 8.

### 3.4. Molecular Docking Analysis

As can be found from the PPI interaction analysis diagram, NTRK1, ESR1, CDK2, CUL3, and TP53 were the proteins with the highest degree values, which were also selected as our core target proteins. We listed the basic information of the target protein and the binding energy of the intrinsic ligand and the protein given in Table 4 (CUL3 had no intrinsic small ligand, so its binding energy was empty). The binding energies of each component to each target protein were listed in Table 5. The target proteins with the best binding energy were given in Table 6, and the number of hydrogen bonds formed was also recorded. The molecular docking results were presented in Figure 9. The binding energy of estrone with CDK2 was −5.9 kcal/mol. As can be seen from Figure 9, the residues THR-14, THR-158, and estrone formed two hydrogen bonds. Estrone and ILE-35, PRO-45, and PHE-152 formed alkyl interactions (Figure 9(a)). The binding energy of 17-beta-estradiol with NTRK1 was −5.5 kcal/mol. There was no hydrogen bond formed between 17-beta-estradiol with NTRK1. The residue ARG-574 and 17-beta-estradiol formed one Pi-alkyl interaction. 17-Beta-estradiol and HIS-503, LEU-532, and GLN-568 formed alkyl interactions (Figure 9(b)). The binding energy between alpha-estradiol and TP53 was −6.85 kcal/mol. LYS-164 of TP53 and alpha-estradiol formed a hydrogen bond. Alpha-estradiol and GLN-100, SER-166, and Mer-169 formed alkyl interactions. Alpha-estradiol and the residue GLN-167 formed one Pi-alkyl interaction (Figure 9(c)). The binding energy of estrone with CUL3 was −4.42 kcal/mol. CUL3 and the residues SER270 and PRO259 formed two hydrogen bonds. The residues ARG266, VAL263, and estrone formed two Pi-cation bonds. Estrone and the residues PRO307 and GLU258 formed alkyl interactions (Figure 9(d)). The binding energy between estrone and ESR1 was −6.46 kcal/mol. Estrone and the residue TYP213 formed two Pi-Pi interactions. Estrone and HIS206, GLU210 formed alkyl interactions (Figure 9(e)).

## 4. Discussion

First recorded in the Shen Nong Ben Cao Jing, deer antlers are true bone growth found in pairs on the heads of male deer and are commonly utilized as Chinese medicine to tonify “kidney-yang,” which is believed to have the effect of strengthening the muscles and bones. Modern pharmacology has found through various experimental studies that deer antlers have significant anti-inflammatory and antioxidant effects, which protect osteoblasts, and this may be the mechanism by which deer antlers treat degenerative disc degeneration. However, few studies explored the molecular mechanism of deer antlers in the treatment of IVDD. Through the network pharmacology and molecular docking analysis of deer antlers for the treatment of IVDD, we have made a preliminary exploration of its molecular mechanism.

The mechanisms by which IVDD occurs are complex, and current studies mainly focus on oxidative stress [17], inflammatory irritation [18, 19], nutritional deficiencies [20], and DNA damage [21]. In the screening results of the small molecule active compounds of deer antlers, we found that the active compounds such as estradiol and estrone are all steroid hormones. It has been found that both *α*-estradiol and 17-*β*-estradiol can increase the activity of anti-inflammatory markers such as IL-6 receptors through the action of estrogen receptors, thereby reducing the secretion of inflammatory factors TNF-*α* and IL-6 and inhibiting inflammatory stimulation [22, 23]. It has also been shown that estradiol protects tissues by inhibiting oxidative stress in organ tissues [24, 25]. The specific mechanism of action is through binding to the estrogen receptor. It is particularly noteworthy that some researchers have found that intervertebral discs and their surrounding tissues have a large number of estrogen receptors and that the use of 17-beta-estradiol is effective in slowing down the process of IVDD, which may be a mechanism for the treatment of IVDD with deer antlers [26–28].

All six pathways are crucial to the occurrence of IVDD. The PI3K-Akt signaling pathway plays a critical role in IVDD [29]. After PI3K-Akt activation, it can help promote the apoptosis of nucleus pulposus cells [30]. It was reported by Krupkova that, through promoting Akt phosphorylation, epigallocatechin 3-gallate prevented nucleus pulposus cells from oxidative stress [31]. The thyroid signal pathway is also an important factor. It has been reported that thyroid hormone can regulate microRNAs to induce an antioxidative stress effect [32]. Several studies reported that the Notch signaling pathway can stimulate chondrogenesis and cartilage development, which has an effect on curing IVDD [33]. It is also reported that the activated Notch signaling pathway reduced the growth arrest and apoptosis of nucleus pulposus cells and promoted the regeneration and proliferation of nucleus pulposus cells [34]. The expression of FoxO protein can induce several kinds of antioxidant enzymes and play the role of antioxidation [35, 36]. Alvarez-Garcia O et al. found that IVDD is associated with an obvious decrease in the number of effectors that receive FoxO signals, which affects the expression of FoxO protein [37]. So, we can deduce that Foxo is an important regulatory protein for antiaging and antioxidation. Maintaining the normal expression of FoxO is essential in delaying IVDD. Estrogen secretion can effectively reduce the incidence of IVDD. Some studies have shown that with a reduction in estrogen secretion, postmenopausal women's incidence of IVDD also increased [38]. Other studies have found that the presence of estrogen helps maintain the extracellular matrix [39]. HIF-1 keeps nucleus pulposus cells alive and synthesizes and maintains the extracellular matrix [40]. At the same time, Hif-1 can regulate the stabilization of oxygen by regulating a variety of enzymes [41].

Molecular docking was utilized to determine if the four components had an affinity for the five target proteins. With the results listed, it indicates that these components could bind tightly to the target proteins. Given that the binding affinity of alpha-estradiol on TP53 was slightly lower than the original ligand, we can conclude that estrone on ESR1 had the best docking result. We can speculate that estrone-ESR1 may have a potential antidenaturation effect.

## 5. Conclusion

In summary, we initially explored the molecular mechanism of deer antlers for the treatment of IVDD through network pharmacology and molecular docking in this study, predicting that the key therapeutic mechanism is anti-inflammatory and antioxidant. We also found that estrone showed the best docking results against ESR1 and predicted that it could be used as a potential drug treatment site. Although the effective compounds from this study screen scored highly, it cannot be determined that the remaining compounds are not clinically effective, especially large-molecule compounds such as peptides. Furthermore, experimental validation of the results of this study is still required due to algorithmic limitations and database sources limited to published research reports.

## Figures and Tables

**Figure 1:** Brief flowchart with network pharmacology and molecular docking.

**Figure 2:** Composition-target network diagram. The triangle represents the active compound and the rectangle represents the target site of action.

**Figure 3:** Flowchart of core target screening.

**Figure 4:** Significant bubble diagram of a biological process.

**Figure 5:** Significant bubble diagram of cell components.

**Figure 6:** Significant bubble diagram of a molecular function.

**Figure 7:** KEGG enrichment results.

**Figure 8:** PI3K-Akt signaling pathway diagram.

**Figure 9:** Molecular docking of components with target proteins. (a) Molecular docking of estrone with CDK2. (b) Molecular docking of 17-beta-estradiol with NTRK1. (c) Molecular docking of alpha-estradiol with TP53. (d) Molecular docking of estrone with CUL3. (e) Molecular docking of estrone with ESR1.

**Table 1:** Active ingredients of TCM.

Ingredient ID	Ingredient name
HBIN001991	17-Beta-estradiol
HBIN015508	Alpha-estradiol
HBIN025818	Estragole
HBIN025821	Estrone
HBIN037857	Estrone

**Table 2:** Key targets of TCM.

Compound	Degree
Alpha-estradiol	58
17-Beta-estradiol	55
Estrone	54
Estrone	54
Estragole	17

**Table 3:** 112 hub genes.

Gene name	Gene name	Gene name	Gene name	Gene name	Gene name	Gene name
NTRK1	SIRT7	HNRNPU	MDM2	YWHAG	TUBB	HIST1H4A
ESR1	YWHAZ	HUWE1	YWHAQ	ARRB2	HNRNPK	HIST4H4
CDK2	CAND1	HDAC5	VHL	FUS	NCL	HIST2H4B
CUL3	OBSL1	HNRNPA1	HSPA5	STAU1	ILF3	HIST1H4I
TP53	NPM1	RPA1	RPA2	HDAC2	RPS3	RPS2
MCM2	ITGA4	HIST1H3C	HSPA8	HDAC3	EIF4A3	CUL4A
EGFR	EP300	HIST1H3E	EEF1A1	TARDBP	HIST1H4C	HNRNPM
XPO1	HSP90AB1	HIST1H3I	CREBBP	RPS27A	HIST1H4H	SMARCA4
FN1	HDAC1	HIST1H3G	CUL2	EZH2	HIST1H4B	TUBG1
UBC	CCDC8	HIST1H3J	PARP1	ACTB	HIST1H4E	PABPC1
GRB2	VCP	HIST1H3H	PAN2	XRCC6	HIST1H4L	RPL6
COPS5	BRCA1	HIST1H3B	U2AF2	CUL4B	HIST2H4A	DHX9
CUL7	VCAM1	HIST1H3D	PRKDC	FLNA	HIST1H4D	ILF2
CUL1	EED	HIST1H3A	SUZ12	RPL10	HIST1H4F	RPL5
HSP90AA1	CDC5L	HIST1H3F	CUL5	RACK1	HIST1H4K	RPS8
RNF2	SNW1	EWSR1	YWHAE	H2AFX	HIST1H4J	RAD21

**Table 4:** Basic information of the target protein and the binding energy of the intrinsic ligand.

Target protein	PDB ID	Ligand ID	Binding energy (kcal/mol)
CDK2	2R3R	6SC	−5.83
NTRK1	5JFW	6K2	−12.50
TP53	6GGC	EXN	−9.21
CUL3	6I2M	—	—
ESR1	7B9R	T4Q	−5.23

**Table 5:** The binding energy of each component to each target protein.

Target protein	Estrone	Estragole	Alpha-estradiol	17-Beta-estradiol
CDK2	−5.90	−3.30	−5.12	−5.75
NTRK1	−4.94	−3.23	−4.65	−5.50
TP53	−6.63	−3.45	−6.85	−6.33
CUL3	−4.42	−1.85	−3.02	−4.16
ESR1	−6.46	−2.94	−5.32	−5.66

**Table 6:** Target proteins with the best binding energy.

Target protein	Component	Binding energy (kcal/mol)	Number of hydrogen bonds
CDK2	Estrone	−5.90	2
NTRK1	17-Beta-estradiol	−5.50	0
TP53	Alpha-estradiol	−6.85	1
CUL3	Estrone	−4.42	2
ESR1	Estrone	−6.46	0

## Data Availability

The data used to support the conclusions of this study are available from the corresponding author upon request.

## Abbreviations

IVDD: Intervertebral disc degeneration
TCMSP: Traditional Chinese medicine systems pharmacology
PPI: Protein-protein interaction
GO: Gene ontology
KEGG: Kyoto Encyclopedia of Genes and Genomes
TCM: Traditional Chinese medicine.

## References

[1] Feleke M., Bennett S., Chen J., Hu X., Williams D., Xu J. (2021). New physiological insights into the phenomena of deer antler: a unique model for skeletal tissue regeneration. *Journal of Orthopaedic Translation*.

[2] Fung F. Y., Linn Y. C. (2017). Steroids in traditional Chinese medicine: what is the evidence?. *Singapore Medical Journal*.

[3] Yao B., Zhang M., Leng X. (2018). Antler extracts stimulate chondrocyte proliferation and possess potent anti-oxidative, anti-inflammatory, and immune-modulatory properties. *In Vitro Cellular & Developmental Biology—Animal*.

[4] Oh C. D., Im H. J., Suh J., Chee A., An H., Chen D. (2016). Rho-associated kinase inhibitor immortalizes rat nucleus pulposus and annulus fibrosus cells: establishment of intervertebral disc cell lines with novel approaches. *Spine*.

[5] Cheung K. M. C., Karppinen J., Chan D. (2009). Prevalence and pattern of lumbar magnetic resonance imaging changes in a population study of one thousand forty-three individuals. *Spine*.

[6] Wu P. H., Kim H. S., Jang I. T. (2020). Intervertebral disc diseases part 2: a review of the current diagnostic and treatment strategies for intervertebral disc disease. *International Journal of Molecular Sciences*.

[7] Teraguchi M., Yoshimura N., Hashizume H. (2017). Progression, incidence, and risk factors for intervertebral disc degeneration in a longitudinal population-based cohort: the Wakayama Spine Study. *Osteoarthritis and Cartilage*.

[8] Ding Y., Ko S. C., Moon S. H., Lee S. H. (2019). Protective effects of novel antioxidant peptide purified from alcalase hydrolysate of velvet antler against oxidative stress in chang liver cells in vitro and in a zebrafish model in vivo. *International Journal of Molecular Sciences*.

[9] Chunhui Y., Wenjun C., Hui W. (2017). Pilose antler peptide protects osteoblasts from inflammatory and oxidative injury through EGF/EGFR signaling. *International Journal of Biological Macromolecules*.

[10] Liu G., Ma C., Wang P. (2017). Pilose antler peptide potentiates osteoblast differentiation and inhibits osteoclastogenesis via manipulating the NF-*κ*B pathway. *Biochemical and Biophysical Research Communications*.

[11] Dong Y., Liu L., Shan X. (2018). Pilose antler peptide attenuates LPS-induced inflammatory reaction. *International Journal of Biological Macromolecules*.

[12] Wang X., Li H., Liu Y. (2020). Velvet antler methanol extracts (MEs) protects against oxidative stress in caenorhabditis elegans by SKN-1. *Biomedicine & Pharmacotherapy*.

[13] Niu B., Zhang H., Li C. (2019). Network pharmacology study on the active components of Pterocypsela elata and the mechanism of their effect against cerebral ischemia. *Drug Design, Development and Therapy*.

[14] Luo T. T., Lu Y., Yan S. K., Xiao X., Rong X. L., Guo J. (2020). Network pharmacology in research of Chinese medicine formula: methodology, application and prospective. *Chinese Journal of Integrative Medicine*.

[15] Zhang R., Zhu X., Bai H., Ning K. (2019). Network pharmacology databases for traditional Chinese medicine: review and assessment. *Frontiers in Pharmacology*.

[16] Morris G. M., Lim-Wilby M. (2008). Molecular docking. *Methods in Molecular Biology*.

[17] Zhang G. Z., Deng Y. J., Xie Q. Q. (2020). Sirtuins and intervertebral disc degeneration: roles in inflammation, oxidative stress, and mitochondrial function. *Clinica Chimica Acta*.

[18] Cazzanelli P., Wuertz-Kozak K. (2020). MicroRNAs in intervertebral disc degeneration, apoptosis, inflammation, and mechanobiology. *International Journal of Molecular Sciences*.

[19] Wang Y., Che M., Xin J., Zheng Z., Li J., Zhang S. (2020). The role of IL-1*β* and TNF-*α* in intervertebral disc degeneration. *Biomedicine & Pharmacotherapy*.

[20] Urban J. P., Smith S., Fairbank J. C. (2004). Nutrition of the intervertebral disc. *Spine*.

[21] Schmitt C. A., Fridman J. S., Yang M. (2002). A senescence program controlled by p53 and p16INK4a contributes to the outcome of cancer therapy. *Cell*.

[22] Santos R. S., de Fatima L. A., Frank A. P., Carneiro E. M., Clegg D. J. (2017). The effects of 17 alpha-estradiol to inhibit inflammation in vitro. *Biology of Sex Differences*.

[23] Debarba L. K., Jayarathne H. S. M., Miller R. A., Garratt M., Sadagurski M. (2022). 17-alpha-Estradiol has sex-specific effects on neuroinflammation that are partly reversed by gonadectomy. *Journals of Gerontology: Series A*.

[24] Khan M., Ullah R., Rehman S. U. (2019). 17*β*-estradiol modulates SIRT1 and halts oxidative stress-mediated cognitive impairment in a male aging mouse model. *Cells*.

[25] Feng D. D., Zheng B., Yu J. (2021). 17*β*-estradiol inhibits proliferation and oxidative stress in vascular smooth muscle cells by upregulating BHLHE40 expression. *Front Cardiovasc Med*.

[26] Wang H., Li Z., Huo Y. (2021). 17*β*-estradiol alleviates intervertebral disc degeneration by inhibiting NF-*κ*B signal pathway. *Life Sciences*.

[27] Li P., Gan Y., Xu Y. (2017). 17beta-estradiol attenuates TNF-*α*-Induced premature senescence of nucleus pulposus cells through regulating the ROS/NF-*κ*B pathway. *International Journal of Biological Sciences*.

[28] Song X. X., Shi S., Guo Z., Li X. F., Yu B. W. (2017). Estrogen receptors involvement in intervertebral discogenic pain of the elderly women: colocalization and correlation with the expression of Substance P in nucleus pulposus. *Oncotarget*.

[29] Liu W., Niu F., Sha H. (2020). Apelin-13/APJ system delays intervertebral disc degeneration by activating the PI3K/AKT signaling pathway. *European Review for Medical and Pharmacological Sciences*.

[30] Yu X., Li Z., Shen J. (2013). MicroRNA-10b promotes nucleus pulposus cell proliferation through RhoC-Akt pathway by targeting HOXD10 in intervetebral disc degeneration. *PLoS One*.

[31] Krupkova O., Handa J., Hlavna M. (2016). The natural polyphenol Epigallocatechin gallate protects intervertebral disc cells from oxidative stress. *Oxidative Medicine and Cellular Longevity*.

[32] Huang P. S., Wang C. S., Yeh C. T., Lin K. H. (2019). Roles of thyroid hormone-associated microRNAs affecting oxidative stress in human hepatocellular carcinoma. *International Journal of Molecular Sciences*.

[33] Haller R., Schwanbeck R., Martini S. (2012). Notch1 signaling regulates chondrogenic lineage determination through Sox9 activation. *Cell Death & Differentiation*.

[34] Long J., Wang X., Du X. (2019). JAG2/Notch2 inhibits intervertebral disc degeneration by modulating cell proliferation, apoptosis, and extracellular matrix. *Arthritis Research and Therapy*.

[35] Nemoto S., Finkel T. (2002). Redox regulation of forkhead proteins through a p66shc-dependent signaling pathway. *Science*.

[36] Kops G. J. P. L., Dansen T. B., Polderman P. E. (2002). Forkhead transcription factor FOXO3a protects quiescent cells from oxidative stress. *Nature*.

[37] Alvarez-Garcia O., Matsuzaki T., Olmer M., Masuda K., Lotz M. K. (2017). Age-related reduction in the expression of FOXO transcription factors and correlations with intervertebral disc degeneration. *Journal of Orthopaedic Research*.

[38] Wang Y. X. J. (2015). Postmenopausal Chinese women show accelerated lumbar disc degeneration compared with Chinese men. *Journal of Orthopaedic Translation*.

[39] Liu Q., Wang X., Hua Y. (2019). Estrogen deficiency exacerbates intervertebral disc degeneration induced by spinal instability in rats. *Spine*.

[40] Wu W. J., Zhang X. K., Zheng X. F., Yang Y. H., Jiang S. D., Jiang L. S. (2013). SHH-dependent knockout of HIF-1 alpha accelerates the degenerative process in mouse intervertebral disc. *International Journal of Immunopathology & Pharmacology*.

[41] Chen S., Fang X. Q., Wang Q. (2016). PHD/HIF-1 upregulates CA12 to protect against degenerative disc disease: a human sample, in vitro and ex vivo study. *Laboratory Investigation*.

